The article "Effect of Virtual Reality on Functional Ankle Instability Rehabilitation: A Systematic Review" was retracted in 2023. Reasons: unreliable results or conclusions; concerns about the data; concerns about the peer review; concerns about the citations.

# Effect of Virtual Reality on Functional Ankle Instability Rehabilitation: A Systematic Review

**DOI:** 10.1155/2021/7363403

**Published:** 2021-11-29

**Authors:** Hongyuan Lin, Kaiyue Han, Bing Ruan

**Affiliations:** ^1^School of Sports Medicine and Rehabilitation, Beijing Sport University, Beijing 100084, China; ^2^School of Rehabilitation Medicine, Capital Medical University, Beijing 100068, China

## Abstract

**Objective:**

To systematically evaluate the effectiveness of virtual reality (VR) in the rehabilitation of patients with functional ankle instability (FAI).

**Methods:**

Nine databases were researched, including PubMed, Cochrane Library, Web of Science, Embase, OVID, CNKI, VIP, WanFang, SinoMed, ResearchGate, and WorldWildScience. The publication date deadline was May 22, 2021. To analyze the effect of VR rehabilitation of FAI, we systematically reviewed the literature using the RevMan 5.4 software. *Main Results.* Five randomized controlled trials (RCTs) were included in the analysis, consisting of 137 patients with FAI; 68 of them were in the experimental group, 69 were in the control group, and all were university students. A comparison study was conducted between the two groups in terms of balance function, muscle performance, and proprioception. VR rehabilitation in the treatment of FAI was found to be significantly more effective using a 30-second single-leg standing test than conventional rehabilitation. The angular offset index of VR rehabilitation training was significantly lower than that of conventional balance training (0.66 ± 0.18 vs. 0.95 ± 0.21; *P* = 0.005).

**Conclusion:**

VR rehabilitation is effective at treating FAI. However, RCTs with higher homogeneity are needed to provide a more reliable evidence-based foundation for clinical rehabilitation.

## 1. Introduction

The ankle is the most commonly injured joint in sports injuries, accounting for 10% to 30% of sports injuries [1]. A significant ankle sprain can lead to loss of proprioception, decreasing muscle strength, and decreased neuromuscular and postural control ability. Without prompt and proper management, a sprain can have serious sequelae, such as ongoing ankle sensory instability and recurrence of the twist [2, 3]. About 32% to 47% of patients with ankle injuries may develop functional ankle instability (FAI) [4]. FAI refers to the patient's subjective belief that the ankle is “softening” or the occurrence of frequent ankle sprains in daily life [5], leading to difficulties for patients in social participation. According to the recommendations from the International Ankle Consortium (IAC), a score ≤ 23 in the Cumberland Ankle Instability Tool (CAIT) is used as the criteria for diagnosing patients with FAI [6]. At present, conventional rehabilitation training for FAI mainly focuses on strength [7, 8], balance [9, 10], proprioception [11, 12], and muscle strength combined with proprioception training [13, 14]. Active functional rehabilitation training in these fields has certain positive effects on ankle stability and postural control ability, but the rehabilitation mode of patients during training is passive, lacks immediate feedback, and cannot stimulate patient's self-efficacy and motivation for actively participating. To address these issues for patients with FAI, the use of virtual reality (VR) rehabilitation has become a research hotspot in recent years.

Due to the global outbreak of COVID-19, there is an increasing trend in noncontact intervention models, such as telemedicine and telerehabilitation [15]. In such an environment, VR rehabilitation training is undoubtedly a more appropriate choice for patients with FAI who need both independent space and goal-oriented movement. VR rehabilitation training is a method that combines rehabilitation training with VR, in which training programs are accomplished for patients by immersing them in a simulated environment [16–18] that is primarily characterized through interactivity and immersive [19]. At present, this method has been widely applied with good reliability and validity in the rehabilitation of patients with neurological injuries, such as stroke [20, 21] and cerebral palsy [22, 23]. However, there are a limited number of studies on the application of this method in patients with FAI, and no systematic review has been conducted. Therefore, this study aims to systematically evaluate the currently published literature on the application of VR rehabilitation in patients with FAI, so as to provide a theoretical basis for its promotion in clinical rehabilitation.

## 2. Materials and Methods

### 2.1. Search Strategy

Nine databases were searched, including PubMed, Cochrane Library, Web of Science, Embase, OVID, CNKI, VIP, WanFang, SinoMed, ResearchGate, and WorldWildScience. The publication date deadline for literature retrieval was May 22, 2021. The search was carried out by combining subject terms with free terms, and the English search terms included “virtual reality,” “virtual reality exposure therapy,” “VR,” “virtual environment,” “on computer,” “simulator,” “game,” “Kinect,” “Nintendo,” “Wii,” “PlayStation,” “X-box,” “ankle instability,” “ankle sprain,” “recurrent sprain,” “chronic ankle instability,” “functional ankle instability,” and “mechanical ankle instability,” while the Chinese terms included “virtual reality,” “virtual reality technology,” “VR,” “virtual rehabilitation,” “virtual environment,” “interactivity,” “virtual world,” “virtual space,” “virtual device,” “gamification,” “ankle instability,” “lateral ankle instability,” “recurrent ankle sprain,” “chronic ankle instability,” “functional ankle instability,” and “mechanical ankle instability.” Meanwhile, the gray literature was searched by tracking the references of the relevant studies and conducting manual retrieval. By taking PubMed as an example, the specific retrieval strategy is shown in Table 1.

### 2.2. Selection of Studies

A double-person extraction method was adopted. Two authors (HY and KY) independently completed literature screening, data extraction, and cross-checking of results. First, the titles and abstract contents were read for preliminary screening, and then, the full texts were read to determine whether the literature met the inclusion criteria. The Korean studies were translated into English by professional translators in related fields, followed by reading of the full text and extracting the data. If any discrepancies were encountered, they were discussed and solved by contacting the corresponding author (B.).

The extracted data information included the following: ① basic information, such as first author, title, and publication date; ② research characteristics, such as research source, number of samples, gender and age of subjects, intervention methods, and intervention periods; ③ implementation of random scheme and blinding method; ④ outcome indicators. If RCTs involved multiple groups of study, only the group data related to the research content were selected, and finally the detailed information was tabulated.

#### 2.2.1. Inclusion Criteria

The following inclusion criteria were used for inclusion from the analysis: ① subjects were patients with FAI; ② interventions included experimental groups that adopted VR rehabilitation alone or rehabilitation training combined with other intervention methods; ③ control measures, such as the control group being treated with other intervention methods without VR rehabilitation training; ④ outcome indicators, including balance function test (e.g., Y-balance test, 30-second single-leg standing balance test, Romberg's test, 15-second single-leg standing balance test, and 60-second standing balance test), muscle strength tests (e.g., isokinetic muscle strength, countermovement jump with arm swing (CMJA) and stance long jump (SLJ)), and proprioceptive function tests (e.g., ankle proprioceptive function); ⑤ study design, including RCTs of patients with FAI treated by VR rehabilitation, in any language.

#### 2.2.2. Exclusion Criteria

The following exclusion criteria were used for exclusion from the analysis: ① non-RCTs, such as case reports, reviews, cohort studies, and cross-sectional studies; ② intervention means or outcome indicators that do not meet the inclusion criteria; ③ unpublished studies, such as dissertations and conference papers; ④ RCTs with difficulties in acquiring complete data; ⑤ phased or repeated studies.

### 2.3. Evaluation of Included Studies

The Cochrane Systematic Review Manual 6.2.0 [24] was used for evaluation, and the results were included in the risk of bias of the RCTs. The specific contents of evaluation included ① generation of random sequence; ② allocation concealment; ③ whether to blind the outcome evaluators; ④ complete outcome data; ⑤ findings of selective reports; ⑥ other sources of bias. Each item was divided into three levels: “high risk,” “low risk,” or “unclear.” RevMan 5.4 software was used to determine quality bias for the included studies.

The improved JADAD scale was used to conduct the assessment on the quality of the included studies. A modified JADAD measure was used to grade the evaluations of included studies depending on random order generation, allocation scheme concealment, randomization and blinding, and presence or absence of depiction of data on details of the withdrawal of individual subjects from the study. A score of 4–7 was classified as a high-quality study and a score of 1–3 as a low-quality study. The improved JADAD rating scale was used to eliminate experimental studies with low quality and ensure the quality of the analysis. Similarly, the quality of the studies was independently evaluated by the two authors (HY and KY). In case any discrepancies were encountered in the results, they were discussed and solved by contacting the corresponding author (B.).

### 2.4. Data Extraction and Synthesis

In this study, Cochrane Review Manager (version 5.4) software was used to analyze statistical heterogeneity. According to the Cochrane Systematic Review Manual 6.2.0, continuous variables were used, and standard mean difference (SMD) and 95% confidence intervals (CI) were used for expressing the data. The test level *α* was set at 0.05. A chi-square (*χ*^2^) test was used to determine whether there was heterogeneity among studies. Statistical heterogeneity was assessed by calculation of the I^2^ statistic of studies with similar comparison treatment groups. When values of *P* ≥ 0.05 and *I*^2^ ≤ 50% were observed, this indicated that there was homogeneity among the studies and fixed effects models were used. On the contrary, if heterogeneity was detected among the studies, random effects models were adopted.

If the results of the included studies showed significant statistical heterogeneity, or the *χ*^2^ test could not be performed due to significant heterogeneity or there was a lack of data, the meta-analysis method was not adopted; instead, the subgroup analysis method was used for systematic evaluation. Results for each outcome measures were considered to be statistically significant if a *P* value was less than 0.05 for the between group comparison.

## 3. Results

### 3.1. Search Results

When the databases were initially searched, 67 relevant studies were obtained, which consisted of 63 in English, four in Korean, and zero in Chinese. When the duplicated publications were removed, this resulted in 45 studies. After reading the titles and abstracts, 21 articles were studies. After further analysis and reading of the full text, and after the selection by inclusion and exclusion criteria, five articles were included for the meta-analysis, including two studies in English and three studies in any of the Korean languages. A flowchart of the literature retrieval strategy is shown in Figure 1.

### 3.2. Description of the Included Studies

A total of 137 subjects with FAI from the five studies were included in the analysis, including 68 subjects in the experimental group and 69 subjects in the control group, all of whom were college students. Of the five intervention groups, two used a Nintendo Wii Fit Plus as a VR device; the other three used VR Box, VR BOSS + mobile APP (Rope Crossing Adventure VR), and Balance Trainer. The control groups underwent conventional rehabilitation training with rehabilitation devices. The specific characteristics of the studies included in the analysis are shown in Table 2.

### 3.3. Methodological Quality

The quality of the included studies was assessed according to the quality evaluation criteria recommended by the Cochrane Systematic Review Manual [24]. All five included studies adopted the methods of randomization and allocation concealment, two of them described the specific randomization method, one described the allocation concealment, and one study explicitly stated the application of single blinding. Four studies included a complete set of results, and the remaining study described the results or the reasons for missing data. The research results were completely reported in all five studies. The risk of bias assessments of the included studies is shown in Figures 2 and 3.

According to the quality test of the improved JADAD scale, two of the five studies scored six points, three scored four points, and all five were considered high-quality studies. The study quality evaluation is shown in Table 3.

### 3.4. Heterogeneity of Included Studies

For the purpose of this study, all the RCTs showed clinical heterogeneity with regard to subjects, interventions, and outcome assessment. While all the RCTs had subjects who met the inclusion criteria for FAI subjects, individual CAIT scores between the studies were significantly different. In terms of interventions, there were significant differences among the VR experimental groups in their approaches to rehabilitation training in terms of specialized instruments used, frequency of intervention, levels of supervision, and availability of instruction.

In terms of outcome indicators, *χ*^2^ test of muscle strength and proprioception could not be carried out due to the large clinical heterogeneity or a lack of data. In terms of statistical heterogeneity, the balance function-related tests were included in this study, and *χ*2 test results were I^2^ = 89%, *P* = 0.02 (Figure 4), indicating significant statistical heterogeneity. According to the previously mentioned results, a meta-analysis was not suitable for this study, so a subgroup analysis was performed for systematic evaluation of the studies.

### 3.5. Balance Function Rehabilitation

#### 3.5.1. Static Balance Test

*(1) Standing Balance Test with Eyes Open*. Four high-quality RCTs reported the results of a standing balance test with eyes open [25–28]: one RCT [25] used the Biodex Balance System (BMS, Shirley, USA), which was reflected in the deviation angle (°) of a plantar balance device to test the stability limit of the patient in a 30-second single-leg standing balance; one RCT [26] used the Biorescue (RM Ingenierie, France) to test the deviation angle (°) when balancing on one leg for 30 seconds; one RCT [27] used Biorescue (RM Ingenierie, France) to test the movement distance (cm) and speed (cm/s) of plantar pressure center while standing on one leg for 15 seconds; one RCT [28] used Biorescue (RM Ingenierie, France) to test the stability limit (cm^2^), movement distance (cm), and movement area (cm^2^) of plantar pressure center during the 60-second balance test.

According to the analysis of the results, two studies [26, 27] used VR headset display devices (immersive VR) for rehabilitation training. Compared to the nonworn VR-HMD device (VR-box; Max, China), wearing the VR-HMD on an unstable support surface (Jumper, Togu, Germany) on both feet for three weeks of balance training significantly affected the length of center of pressure (COP) during 30-second single balance tests, which showed statistically significantly differences across groups (*P* < 0.05) [26]. By comparing the studies in which subjects wore VR BOSS headset devices combined with mobile integrated VR devices and conventional standing balance training, the speed and length of COP during 15-second single-leg standing balance test improved significantly in both groups after training as compared to before. However, there were no significant differences in these outcomes between the virtual reality training group and the conventional balance training group (*P* > 0.05) [27]. These results suggest that further investigation is required to determine whether the use of VR headsets for rehabilitation training is more effective than conventional balance training in improving ankle instability.

Two studies [25, 28] used VR plane display devices (desktop VR) for rehabilitation training. one high-quality RCT [25] showed that the four-week muscle strength and balance training using VR (Nintendo Wii Fit Plus) improved static balance with a significantly lower angle deviation index (0.66 ± 0.18) during the 30-second single-leg standing balance test on a platform (Biodex Balance System, BMS, Shirley, USA) than that of conventional strength and balance training (0.95 ± 0.21; *P* = 0.005). No significant differences were found in the anterior–posterior (AP) and medial–lateral (ML) directions between the two groups (*P* > 0.05). In terms of the dynamic balance data results on ML direction of level 2 ML (*P* = 0.010), level 4 ML (*P* = 0.016), and level 8 ML (*P* = 0.002), during 30-second single-leg standing balance test on a platform with adjustable unstable levels (Biodex Balance System, BMS, Shirley, USA), the angle deviation index in the VR rehabilitation training group was also significantly lower than that of the conventional strength and balance training group. No significant differences were found in the overall and AP directions between the two groups (*P* > 0.05). This indicates that, compared with conventional training with strength and balance rehabilitation devices, VR rehabilitation training combined with a Nintendo Wii Fit Plus yields better resultes in improving ankle static and dynamic stability. By also comparing the use of treadmill training and VR postural adjustment fusion training with the balance trainer and aero-step, we found a reduction in the 60-second standing balance test in the area of foot pressure movement (*P* < 0.05), the distance moved (*P* < 0.001), and an increase in the stability limit (*P* < 0.05) in the VR group, thus indicating a significant increase of the plantar center of pressure control. The differences in these indicators between the VR-based training group and the treadmill training group were statistically significant [28]. These results indicate that rehabilitation training assisted by a VR plane display device is superior to conventional strength, balance, and treadmill training for improving ankle joint stability. However, this conclusion needs to be confirmed by future studies.

*(2) Romberg*. '*s Test*. One high-quality RCT [26] reported the results of Romberg's test using Biorescue (RM Ingenierie, France), in which the subjects stand upright, put their legs together, and extend their upper limbs forward, for 60 seconds while closing and opening their eyes, respectively, and the outcome indicator is expressed as the distance (cm) of plantar pressure center movement. The results showed that, compared with the NUS group (non-VR-HMD + unstable surface group), the VUS group (VR-HMD + unstable surface group) exhibited a clear and statistically significant improvement in ankle stability (*P* < 0.05).

#### 3.5.2. Dynamic Balance Test (Y-Balance Test)

One high-quality RCT [26] reported the results of a Y-balance test using a Biorescue (RM Ingenierie, France) and presented the results as the sum of the furthest movement distance (cm) of the subject's second toe in the three directions of front, back outside, and back inside. The results showed that the VUS group trained on an unstable support base displayed a more significant improvement in dynamic ankle sympathetic balance compared with the NUS group, and the differences were statistically significant (*P* < 0.05).

### 3.6. Muscle Strength Rehabilitation

#### 3.6.1. Isokinetic Muscle Strength Test

Two high-quality RCTs [26, 29] reported the results of the isokinetic force test, both using a Biodex isokinetic force meter (BMS, Shirley, USA), to test peak torque (N•m). One of the RCTs [26] compared the change rate of muscle strength in four directions (ankle inversion, eversion, plantar flexion, and dorsi flexion) in the VUS and NUS groups before and after training. The results showed that the VUS group exhibited a more significant improvement in muscle strength of the ankle joints in four directions than the NUS group, and the difference was statistically significant (*P* < 0.05). In addition, the results of another RCT [29] confirmed that, compared with conventional strength balance training (TRI group), muscle and balance training using a Nintendo Wii Fit Plus combined with VR (virtual reality assisted intervention (VRAI) group) had no significant advantages in improving strength in the four directions, and the difference between groups was not statistically significant (*P* > 0.05).

#### 3.6.2. Jump Test

A high-quality RCT [28] evaluated that the height (cm) of CMJA and distance (cm) of SLJ using G-Jump (IBTS Bioengineering, Italy). The results showed that, compared with the training on treadmills, the VR posture adjustment fusion training using the balance trainer and aero-step had a more obvious effect on improving the performance of indexes reflecting muscle strength, such as CMJA and SLJ, and the difference was statistically significant (*P* < 0.001).

### 3.7. Proprioception Rehabilitation

One high-quality RCT [26] reported the results of the ankle proprioception test, and the outcome indicators were expressed as the difference between a fixed angle and self-perceived angle (°). The results showed that, compared with the NUS group, the change of proprioception correct angle before and after ankle joint training decreased significantly in the VUS group, and the difference was statistically significant (*P* < 0.05).

## 4. Discussion

In addition to mechanical ankle instability from damage to ankle structures, in accordance with data from epidemiological surveys, more than 60% of chronic ankle instability (CAI) is accounted for by FAI [30]. It is likely that FAI may cause significant problems for patients' social participation, such as reduction in physical activity, stair climbing, and taking part in leisure activities, which can have a negative impact on a person's daily life [31]. In recent years, the use of VR rehabilitation has increased gradually [32]. VR rehabilitation not only improves the patient's participation interest, but also converts patients from passively receiving to actively participating in treatment. In addition, VR rehabilitation improves patient treatment compliance, fully mobilizes all human and material resources needed for training, and improves the efficacy of the training. Additionally, since the VR system is used at home, it can be considered beneficial for the continuous rehabilitation management of patients in the long run [33].

In the current study, in addition to the five RCTs included in the analysis, there were six other RCTs [34–40] that also assessed the feasibility of VR in the rehabilitation of patients with FAI. The six RCTs all adopted the Nintendo Wii Fit Plus for VR rehabilitation training. The studies showed that VR rehabilitation training can improve the static balance [34, 35], dynamic balance [34], proprioception, CAIT score [36], and muscle strength [37] of patients with FAI, and VR balance training may show better results than conventional strength training [38]. However, other studies have reported [39] that, compared with rehabilitation training without any VR interventions, rehabilitation training by VR combined with Kinesio tape does not improve the static and dynamic balance function of patients with FAI in the overall, AP, and ML directions. Other studies suggest that VR rehabilitation training should be performed after the application of Kinesio tape and microwave diathermy therapy [40], but the specific efficacy of this approach remains to be explored further [35].

Based on the five included RCTs on rehabilitation training of patients with FAI, this study summarized the effects of VR rehabilitation on balance function, proprioception, and muscle strength. The results showed that the effect of VR rehabilitation training on improving ankle function, in terms of ankle proprioception [26], Y-balance test [26], 30-second single-leg standing balance test [26], Romberg's test [26], 60-second standing balance test [28], CMJA [28], SLJ [28], and other indicators, is significantly better than that of conventional balance training or treadmill training.

As for the standing balance [25, 27] and isokinetic muscle strength [29] functional tests, three studies reported no differences between VR and conventional exercise, and the possible reasons were analyzed as follows.

According to the study [25] that used VR (Nintendo Wii Fit Plus) and conventional rehabilitation for the four-week muscle strength and balance training to improve balance function, no significant differences were found in the deviation angle (°) of the AP and ML directions of static balance between the two groups, and also no significant differences were found in the overall and AP directions of dynamic balance between the two groups. Questions exist as to why only some parameters were affected after the exercises, and the most plausible reason is the short intervention period (only four weeks) since there appears to be an overall trend towards improvement in balance even though no significant differences were found in some of the analyzed parameters.

According to another study [27] that used the Biorescue (RM Ingenierie, France) device to test the distance (cm) and speed (cm/s) of plantar pressure center movement when subjects balanced on one leg for 15 seconds, compared with conventional standing balance training, the use of VR BOSS headsets combined with mobile integrated VR devices in balance training also had no significant therapeutic advantages in reducing the distance and speed of plantar pressure center movement, thus indicating no significant increase of the plantar center of pressure control in the VR group. The possible explanations for this observation are as follows: first, the training frequency and intensity were the same between the two groups; second, the training program was not individualized and the difficulty was not adjusted according to the unique conditions of each research subject; lastly, four weeks of training time was too short of a duration.

In two studies [26, 29], the peak torque (N•m) of isokinetic force was measured using the Biodex Isokinetic Force Meter (BMS, Shirley, USA) VR device, with different results. One of the RCTs [29] showed no significant difference between the intervention and control groups in the isokinetic muscle strength test, indicating that, compared with the TRI group, the VRAI group had no obvious advantage in improving muscle strength in the four directions of ankle inversion, eversion, plantar flexion, and dorsi flexion. There are two possible reasons to explain this observation. First, the training program for the VRAI group was originally developed for personal leisure exercise, which may not be sufficient to meet the demands of ankle rehabilitation training. Second, conventional rehabilitation usually focuses on specific joints with structural resistance movement, whereas the VRAI group's training content was based on controlling ankle movement by standing on the Wii Fit game board, mainly for training plantar flexion.

Regarding the RCTs included in this study, we found that there were relatively few RCTs on the efficacy of VR rehabilitation for patients with FAI. Also, there is a lack of unified criteria for the inclusion of study objects, and most clinicians take the scores of the functional questionnaire as the assessment standard for FAI patients. In this study, the four included RCTs [25, 27–29] used CAIT to assess the ankle function of patients, three of which [25, 27, 28] considered CAIT scores <24 as the criteria for inclusion of FAI patients, while another RCT [29] used CAIT scores ≤24. Another included RCT [26] chose the Functional Ankle Instability Questionnaire (FAIQ) as the criteria for inclusion of patients with FAI and five or more of the nine true and false questions in FAIQ should be answered “yes.” As a result, this may have led to baseline differences in the subjects due to the inconsistent inclusion criteria. Meanwhile, the different answers to different questions in the same questionnaire may reflect different dysfunction of the patients which should take into account in the development of future training plan. Although VR rehabilitation training has the advantages of self-interest, autonomy, and sustainability, the current rehabilitation management system still lacks an integrated system. Therefore, due to the lack of standardized training programs and procedures for patients with FAI, it is difficult to coordinate the application of conventional rehabilitation therapy and innovative VR rehabilitation technology for the treatment of FAI. Furthermore, the outcome indicators were difficult to classify and integrate due to the high heterogeneity [25, 26].

Overall, the reviewed clinical trials were limited by the heterogeneity in VR and conventional rehabilitation interventions as well as outcome measures. Thus, comparing different studies and conducting a meta-analysis was not possible. In addition to the outcome indicator data, the material and labor cost of VR and conventional rehabilitation training should also be presented and compared in RCTs studies, or the missing data may result in biases due to the pooling effect [41].

The following four points are our recommendations for improving RCTs studying the efficacy of VR rehabilitation for patients with FAI: first, the duration of the intervention should be extended, the study area should be expanded, the age range of the study objects should be broadened, and a wide range of RCTs should be carried out to obtain relevant data. Second, the inclusion criteria for patients with FAI should be further harmonized and as FAI is primarily determined by self-reported characteristics, it is important that people are able to fully understand, consistently remember, and report these symptoms. Third, the selection of VR rehabilitation interventions should be standardized, and outcome indicators should be unified and should require repeated measurements to minimize heterogeneity. Also, other outcome measures, such as CAIT score, ankle range of motion, and participant satisfaction, might also be clinically important for the evaluation of patients with FAI. Fourth, economic and social benefits should be analyzed in addition to clinical efficacy. Lastly, VR rehabilitation-related technologies, such as biofeedback, augmented reality, gamification, and remote rehabilitation, should be more widely used in studies of VR rehabilitation of FAI.

## 5. Limitations

To our knowledge, this is the first study to systematically review and assess the quality of RCTs investigating the effectiveness of VR in FAI rehabilitation. It is important to note that some limitations exist in this systematic evaluation. First, only five RCTs were included in this study, and the characteristics of the patient baseline indicators were not completely consistent. Second, three of the RCTs included in this study were in Korean, and although they were fully translated by professional translators, there may have been some understanding biases due to the translation or reading. Third, due to the limited number of samples and relatively short intervention time, the final results were inevitably less accurate [42]. Finally, due to the heterogeneity of the study subjects, intervention measures, control measures, and outcome indicators, a meta-analysis could not be performed [43].

## 6. Conclusion

RCTs investigating whether VR can improve the rehabilitation process of patients with FAI are scarce and have not yet been able to draw accurate evidence-based clinical suggestions. In this study, the overall positive effect of VR rehabilitation on improving balance, muscle weakness, and proprioception was better than that of conventional rehabilitation. However, our analysis included a limited number of tests with low-quality methodology, which reduced the reliability of the conclusions to an extent. In the future, high-quality studies with increased homogeneity are needed to provide more reliable evidence-based clinical evidence for the use of VR rehabilitation in the treatment of patients with FAI.

## Figures and Tables

**Figure 1:** Literature search strategy.

**Figure 2:** Risk of bias diagram.

**Figure 3:** Summary of risk of bias in the included studies. “+”: low risk; “—”: high risk; “?”: unclear risk.

**Figure 4:** A forest plot of standardized (std.) mean difference, with 89% confidence interval (89% CI) for FAI measured with balance function-related tests between the virtual reality (VR) and conventional treatment groups. IV: inverse variance.

**Table 1:** Retrieval strategy (using PubMed as an example).

The formulation of retrieval format
(“Virtual reality exposure Therapy”[MeSH terms] OR “virtual Reality”[MeSH terms] OR (“VR”[Title/Abstract] OR “virtual environment”[Title/Abstract] OR “computer-based”[Title/Abstract] OR “simulator”[Title/Abstract] OR “game”[Title/Abstract] OR “gaming”[Title/Abstract] OR “Kinect”[Title/Abstract] OR “Nintendo”[Title/Abstract] OR “Wii”[Title/Abstract] OR “Playstation”[Title/Abstract] OR “X-box”[Title/Abstract])) AND (“ankle instability”[Title/Abstract] OR “ankle unstable”[Title/Abstract] OR “ankle sprain”[Title/Abstract] OR “recurrent sprain”[Title/Abstract] OR “chronic ankle instability”[Title/Abstract] OR “functional ankle instability”[Title/Abstract] OR “mechanical ankle instability”[Title/Abstract]) AND (“randomized controlled trial”[Publication type] OR “randomized”[Title/Abstract] OR “placebo”[Title/Abstract])

**Table 2:** Description of the included studies.

Included studies	Country	Cases		Age/year		VR type	Interventions		Number of Interventions/week	Frequency	Outcome indicators
		VR group	Control group	VR group	Control group		VR group	Control group			
Baek et al. 2019 [26]	South Korea	20	22	20.00-29.00		VR box	5 min warm up and stretch. 20 min VR training: wear VR-HMD (VRbox; Max, China), stand on an unstable support surface (JUMPER; TOGU, Germany) for balance training. 5 min relax and stretch.	5 min warm up and stretch. 20 min conventional training: without VR-HMD, stand on an unstable support surface (JUMPER; TOGU, Germany) on both feet for balance training. 5 min relax and stretch.	3	3 times/week; 20 min/time	①②③④⑤

Kim et al. 2018 [29]	South Korea	10	10	21.80 ± 1.20	22.10 ± 2.40	Nintendo Wii Fit Plus	5 min warm up and stretch. 20 min VR training: muscle strength and balance strengthening exercises with Nintendo Wii Fit Plus.	5 min warm up and stretch. 20 min conventional training: ankle muscle strength training in four directions with elastic bands; stand on the aero step (TOGU, Germany) on one foot in situ for balance training.	4	3 times/week; 20 min/time	②

Kim et al. 2019 [25]	South Korea	10	11	21.00 ± 1.20		Nintendo Wii Fit Plus	5 min warm up and stretch. 20 min VR training: 10 min of muscle strength and 10 min of balance strengthening with Nintendo Wii Fit Plus. 5 min relaxation activities.	5 min warm up and stretch. 20 min conventional training: ankle muscle strength training in four directions with elastic bands; balance training in appropriate difficulty with Airex Balance Pad, slide board, donut hall, trampoline, Bosu Pro Balance Trainer, basic balance board and rocker/wobble board package. 5 min relaxation activities.	4	3 times/week; 20min/time	④
Kim et al. 2020 [27]	South Korea	13	11	21.38 ± 1.00	21.90 ± 1.00	VR BOSS & APP： rope crossing adventure VR	10 min warm up. 30 min VR training: use mobile comprehensive virtual reality trainer VR BOSS (Smpia; Seoul, Republic of Korea) combined with rope crossing adventure VR APP to perform balance training (1-2 weeks of tightrope walking indoors, 3-4 weeks of tightrope walking between high-rise buildings).	10 min warm up. 30 min conventional training: static and dynamic balance training such as open/closed eyes, standing on one foot, knee lifting on one leg, one foot standing squat, etc. (1-2 weeks on the ground /wobble balance boards, 3-4 weeks on the balance pads).	4	3 times/week; 30min/time	⑥

Yang et al. 2016 [28]	South Korea	15	15	21.36 ± 2.92	22.04 ± 4.05	Balance trainer	30 min plyometric training: zigzag running, backward running, vertical jumping, agility jumping, side jumping, full speed running, and other sports. 30 min VR training: VR-based fusion training of neuromuscular postural control: use Aero step (TOGU, Germany) in combination with the Balance trainer (Medica Medizintechink GmbH, Germany) for training.	30 min plyometric training: zigzag running, back running, vertical jump, agility jump, side jump, full speed running. 30 min conventional training: run on treadmill.	8	3 times/week; 30min/time	⑦⑧⑨

① Ankle proprioceptive sense; ② isokinetic muscle strength (Biodex isokinetic force meter; BMS, Shirley, USA); ③ Y-balance test; ④ 30-second single-leg standing balance test (Biorescue; RM Ingenierie, France/Biodex balance system; BMS, Shirley, USA); ⑤ Romberg's test (Biorescue; RM Ingenierie, France); ⑥ 15-second single-leg standing balance test (Biorescue; RM Ingenierie, France); ⑦ 60-second standing balance test (Biorescue; RM Ingenierie, France); ⑧ CMJA (G-jump; IBTS bioengineering, Italy); ⑨ SLJ (G-jump; BTS bioengineering, Italy). CMJA: countermovement jump with arm swing; SLJ: stance long jump;

**Table 3:** Scores from of the improved JADAD study quality evaluation.

	Random sequence generation	Randomized concealment	Blinding	Withdrawal	Score
Baek et al., 2019 [26]	1	1	1	1	4
Kim et al., 2018 [29]	2	1	2	1	6
Kim et al., 2019 [25]	2	2	1	1	6
Kim et al., 2020 [27]	1	1	1	1	4
Yang et al., 2016 [28]	1	1	1	1	4

## Data Availability

All data generated or analyzed during this study are included in this published article.
